The article "Digital image processing technology under backpropagation neural network and K-Means Clustering algorithm on nitrogen utilization rate of Chinese cabbages" was retracted in 2023. Reasons: unreliable results or conclusions; concerns about the peer review.

# Digital image processing technology under backpropagation neural network and K-Means Clustering algorithm on nitrogen utilization rate of Chinese cabbages

**DOI:** 10.1371/journal.pone.0248923

**Published:** 2021-03-31

**Authors:** Qilin Wang, Xinyu Mao, Xiaosan Jiang, Dandan Pei, Xiaohou Shao

**Affiliations:** 1 College of Agricultural Science and Engineering, Hohai University, Nanjing, China; 2 Taizhou Research Institute of Nanjing Agricultural University, Taizhou, China; Ministry of Natural Resources North Sea Bureau, CHINA

## Abstract

The purposes are to monitor the nitrogen utilization efficiency of crops and intelligently evaluate the absorption of nutrients by crops during the production process. The research object is Chinese cabbage. The Chinese cabbage population with different agricultural parameters is constructed through different densities and nitrogen fertilizer application rates based on digital image processing technology, and an estimation NC (Nitrogen Content) model is established. The population is classified through the K-Means Clustering algorithm using the feature extraction method, and the Chinese cabbage population quality BPNN (Backpropagation Neural Network) model is constructed. The nonlinear mapping relationship between different agricultural parameters and population quality, and the contribution rate of each indicator, are studied. The nitrogen utilization of Chinese cabbage is monitored effectively. Results demonstrate that the proposed NC estimation model has correlation coefficients above 0.70 in different growth stages. This model can accurately estimate the NC of the Chinese cabbage population. The results of the Chinese cabbage population quality BPNN model show that the population planting density based on the seedling number is reasonable. The constructed population quality evaluation model has a high R^2^ value and a comparatively low RMSE (Root Mean Square Error) value for the quality evaluation of Chinese cabbage in different periods, showing that it applies to evaluate the population quality of Chinese cabbage in different growth stages. The constructed nitrogen utilization model and quality evaluation model can monitor the nutrient utilization of crops in different growth stages, ascertain the agricultural characteristics of other yield groups in different growth stages, and clarify the performance of agricultural parameters in different growth stages. The above results can provide some ideas for crop growth intelligent detection.

## Introduction

China is an agricultural power, in which agricultural production acts as a vital link between its economic construction and social development. China has the largest area of facility horticulture cultivation [1]. Vegetables play a pivotal role in the national economy, and their contribution to the national economy continues to increase with economic development. The sown area and total output of vegetables accounted for 43% and 49% of the world’s, respectively, ranking the first worldwide [2]. The sown area of vegetables in China increased from 4.7533 million hm^2^ to 17.3287 million hm^2^ from 1985 to 2019, with an average growth rate of 5.79%. In 1989, vegetable production was 176 million tons; by 2018, it increased to 565 million tons; the 20-year average growth rate reached 6.32%. In 2000, the national vegetable sown area was 13.67 million hm^2^, accounting for 35% of the world’s total area. The average annual vegetable per capita was 350kg, which was 100kg higher than the world average.

Moreover, the total vegetable output was 440 million tons, accounting for more than half of the world’s total output, whose value reached 300 billion Chinese yuan. Thus, vegetable has become the second-largest agriculture output in China after food [3]. In provinces such as Shandong and Hebei, the total output value of vegetables has surpassed grain, becoming the largest industry. In 2002, China’s national vegetable sown area reached 19 million hm^2^, the total output exceeded 520 million tons, and the total output value reached 350 billion Chinese yuan. In 2007, the national vegetable sown area approached 17 million hm^2^, the total output reached 565 million tons, and the total output value was 720 billion Chinse yuan.

Furthermore, the sown area of vegetables in autumn and winter alone reached 8.68 million hm^2^ in 2007, with a total output value of 803.9 billion Chinese yuan [4]. In 2019, the output value of China’s facility vegetables accounted for 51% of the national total output value, and the area reached 3.347 million hm^2^, accounting for only 25% of the total vegetable horticulture area. However, as the output of vegetables in China keeps increasing annually, some problems occur in production [5]. In particular, the current technology cannot effectively monitor crops’ growth, which has become an urgent problem in the agricultural field.

At present, facility agriculture has achieved the automatic control of environmental conditions. Y. Hashimoto believed that people should communicate with crops so that crops could change their growth environment according to their growth needs. At present, greenhouses are primarily based on measurement and control technologies, in which the sensors are widely accepted to monitor environmental information factors of facility horticulture and crops’ physiological information [6]. Generally, the monitored greenhouse environmental information principally includes temperature, humidity, carbon dioxide concentration, and light intensity. In the meantime, computer technology, especially image processing technology, is seldom applied to environmental control, water irrigation, crop growth, and pest monitoring. Bengochea et al. (2016) developed a small crop inspection tool based on image processing technology. This method could extract the number of crop rows in real-time from the image acquired by the reflective camera located on the front of the robot under uncontrolled lighting conditions [7]. Mahalakshmi and Shanthakumari (2017) designed an image processing algorithm to identify diseases in rice. The results proved that this image processing technology could more accurately identify diseases and insect pests, helping people decide when to use pesticides to increase crop yields [8]. Dhingra et al. (2018) utilized image processing methods for a comprehensive study on identifying and classification crop leaf diseases. They found that image processing technology could effectively diagnose crop leaf diseases [9]. Vasilaki et al. (2018) applied the clustering analysis method to effectively monitor crop nitrogen uptake [10]. Zhou et al. (2019) used chlorophyll fluorescence images to distinguish different nitrogen processing methods correctly and developed a classification method using chlorophyll fluorescence-induced imaging analysis based on Artificial Neural Networks (ANN) [11]. The above works reveal the feasibility of applying digital image processing technology, Backpropagation Neural Network (BPNN), and clustering analysis to crop monitoring. However, the current research focuses less on the dynamic monitoring of vegetable nutrition, lacking corresponding prediction models as well.

According to the research questions above, a nitrogen concentration model is established through the digital processing technology based on previous research. The application research of digital processing technology in crop nutrition monitoring is considered, in an effort to solve the problem of vegetable nitrogen utilization. The image information of vegetables at different growth stages is extracted from the crop feature data. The K-means Clustering algorithm is used to classify the above information rationally. The BPNN is applied to construct a nonlinear mapping of the quality of the vegetable population and the contribution relationship of each indicator. A timely and accurate diagnosis method for crop nitrogen nutrition is established to determine the scientific fertilization management measures, which are of great significance for improving fertilizer utilization and protecting the environment.

The innovative points are: (1) the application of digital processing technology in crop nitrogen utilization is further refined, and the nitrogen concentration is monitored dynamically. (2) The nitrogen prediction ability of the model is improved through reasonable classification and data learning, which is very crucial for agricultural fertilization. (3) Factors affecting crop growth at different stages are effectively clarified through the quality monitoring of vegetable groups, which has a significant reference value for vegetable quality control.

There are five sections in total. The first section is the introduction, in which the importance of monitoring crop growth is put forward, and the research ideas are determined. The second section is a literature review, in which the research framework is clarified based on the analysis of digital image processing and crop nitrogen determination. The third section is the research method, where the process of experimental planting, nitrogen processing, data acquisition, model construction, and performance evaluation is clarified. Besides, the nitrogen model for Chinese cabbage is constructed. The fourth section provides the results and discussions. The proposed model is tested through specific examples and regression analysis, and its feature evaluation and quality evaluation results are compared with those of previous studies. The fifth section demonstrates the conclusion, including the key results, actual contributions, limitations, and future research directions.

## Literature review

### Digital image processing

Using image analysis technology to measure agricultural parameters directly has good portability and high application value; however, the complexity of the farmland environment and the dynamic variability of crop groups make it difficult to measure various indicators directly. Some agricultural parameters that are difficult to be measured directly are associated with crop image features. Therefore, agricultural parameter estimation models have emerged. Among the research on the estimation models, the nitrogen estimation model is the most extensively accepted. The reason is that nitrogen directly affects the color of crop leaves, while the color feature is the most intuitive and easy to extract feature of the crops’ images.

The color of the crop canopy is closely linked to its nitrogen nutrition status. Therefore, visible light spectrum analysis technology in crop nitrogen nutrition diagnosis has received widespread attention. Especially with the popularity of digital cameras and smartphones, applying digital imaging technology to diagnose the nitrogen nutrition of crops becomes a possibility. Feng et al. (2019) systematically studied the application of digital images in diagnosing wheat nitrogen nutrition. They believed that the angle between the camera and the canopy, the intensity of the sun, the image storage format and resolution, and whether the farmland was irrigated would affect the diagnosis of wheat nitrogen nutrition according to the color parameters of the images [12]. Wang et al. (2020) used a digital camera to take cotton canopy images and found that the green light value (G) and the ratio of green light to red light (G/R) of the image could be used as diagnostic indicators of cotton nitrogen nutrition [13]. Yang et al. (2020) adopted the ratio of green light to blue light (G/B) of digital images to diagnose the nitrogen nutrition of potatoes [14].

### Crop nitrogen determination

At present, methods of using crops’ images for nutritional diagnosis include determination of total nitrogen content of crops, determination of chlorophyll content of crop leaves, and determination of nitrogen content of crop tissue juice. Factors such as soil nutrient status, the crop’s nutrient requirements, and the crop’s ability to absorb nutrients lead to nutritional status differences. Therefore, the measurement of the nutrient factor content in the crop can reflect the current nutritional status of the crop, which can be used to support the fertilization decisions in field management [15]. The diagnosis of crop nitrogen content uses chemical detection methods to judge the abundance or deficiency of nitrogen nutrition. Such a method depends on laboratory chemical analysis to determine the critical concentration of nutrients in different crop organs. The determination of crop total nitrogen content is currently the earliest and most comprehensive indicator that can accurately represent the nitrogen level of crops, which is also correlated with crop yields. The traditional chemical methods to determine the total nitrogen content in crops include Dumar’s method and the Kjeldahl method [16]. The principle of applying Dumar’s method to monitor the nitrogen content of crops is to burn the collected samples to ensure that various forms of nitrogen are converted into gaseous nitrogen; then, the nitrogen content of the samples is calculated by calculating the volume of nitrogen [17]. Almost all the laboratory chemical analysis methods require drying and grinding procedures after collecting crop samples, involving drugs with potential safety hazards. Besides, lots of human and material resources are spent in the experimental process, resulting in poor real-time performances. Besides, laboratory chemical analysis requires experienced professionals, specialized equipment, and chemical reagents, which is difficult for ordinary farmers to master and cannot be promoted on a large scale.

There are many information agriculture applications in previous research, such as agricultural product classification, disease diagnosis, and weed identification. However, practical applications are not involved, which requires further investigation. Besides, a real-time monitoring and nitrogen diagnosis model is the premise of meeting the needs of greenhouse production and “precise” management of Chinese cabbages. Modern computer vision technology can provide systematic analysis and quantitative description of the relationship between the appearance characteristics of Chinese cabbages (leaf color changes) and nitrogen content, establish the mathematical model, simulate the diagnosis of nitrogen, and guide the production, achieving high-quality horticulture and balanced supply of Chinese cabbages.

## Materials and methods

### Digital image processing technology

Modern information technologies adopted for non-destructive monitoring, including satellite remote sensing, near-earth hyperspectral remote sensing, and image analysis, can actively improve crop production management and yield prediction, which is also a vital link to modern agriculture [18]. Digital image analysis uses computers to process graphics or images to obtain valuable information. Then it uses the information obtained to make meaningful decisions. The equipment required includes cameras, digital image collectors, computers, and display terminals, as shown in Fig 1 below [19].

**Fig 1:** A schematic diagram of the image analysis process.

The basis of using image analysis technology to monitor agricultural conditions is the image itself. Commonly used image acquisition devices first obtain RGB (Red, Green, Blue) images, and a series of following operations are performed on RGB images, as shown in Fig 2. An RGB image is an MxNx3 array of color pixels, where each pixel corresponds to the three components of red, green, and blue at a unique spatial location [20]. The first step in using the model to estimate agricultural parameters is to extract image features. Generally, image features include three categories: color feature, texture feature, and morphological feature. Color is the most easily perceivable visual attribute by the human eye. The color feature is a common feature in image analysis. Compared with other features, it is very robust to image rotation changes and translation [21]. The morphological feature is an important indicator to describe the image. It is intuitive and can distinguish crop species or detect crop diseases when the colors are similar. The texture feature is a common visual phenomenon, irregular in part but regular in the whole. There are many texture features in agricultural production [22].

**Fig 2:** A schematic diagram of the RGB color image structure.

### Clustering algorithm and BPNN

The advantages of the K-Mean Clustering algorithm are: (1) the principles are simple, the implementation is easy, and the convergence speed is fast. (2) The clustering effect is better. (3) The interpretability of the algorithm is strong. (4) The parameter that needs to be adjusted is only the cluster number k. The advantages of BPNN are: (1) it has nonlinear mapping capability. BPNN essentially achieves a mapping function from input to output. The mathematical theory proves that a three-layer neural network can approximate any nonlinear continuous function with arbitrary precision. (2) It has self-learning and adaptive capabilities. BPNN can automatically extract the “reasonable rules” between input and output data through learning and adaptively memorize the learned rules in the network weights. The monitoring of crop nitrogen images in agriculture requires low cost, convenience, and feasibility. BPNN is the most straightforward learning network. Hence, these two methods are finally selected for modeling.

1. K-Means Clustering algorithm: it is an unsupervised algorithm that is comparatively uncomplicated to implement and has a better clustering effect; thus, it is widely accepted. It divides a given sample set into *K* clusters according to the distance between the samples. Simultaneously, it makes the clusters’ points as close together as possible and the distance between them as large as possible [23]. In the mathematical expression, assuming that the cluster is divided into *(C*_*1*_, *C*_*2*_, …, *C*_*k*_*)*, the goal is to minimize the squared error *E*:
  $$E=\sum_{i=1}^{k}\sum_{x\in C_{i}}^{k}{\left\|x-u_{i}\right\|}_{2}^{2}$$ (1)
  In (1), *u*_*i*_ refers to the mean vector of the cluster *C*_*i*_, sometimes called the centroid. Its expression is:
  $$u_{i}=\frac{1}{C_{i}}\sum_{x\in C_{i}}^{k}x$$ (2)
  Only the heuristic iterative method can directly find the minimum of the above equation. The K-Means Clustering algorithm should first select a suitable *k* value based on the prior experience of the data through cross-validation. Second, it should select *k* initialized centroids. Because it is a heuristic method, the location of *k* initialized centroids has a significant influence on the final clustering result and running time. Therefore, it is necessary to select the appropriate *k* centroids, and these centroids should not be too close [24].
2. BPNN: it is a multi-layer feedforward network trained according to the error backpropagation algorithm. It is one of the most widely used neural network models for function approximation, model recognition and classification, data compression, and time series forecasting [25]. It has strong self-adaptation, self-learning, and nonlinear mapping capabilities and can solve the problems of less data, insufficient information, and uncertainty. Besides, it is not limited by nonlinear models [26]. A typical BPNN should include three layers: the input layer, hidden layer, and output layer. In this neural network, the calculation of a neuron is as follows:
  $$a_{j}^{l}=\sigma (\sum_{k}w_{jk}^{l}a_{k}^{l-1}+b_{j}^{l})$$ (3)
  In (3), $w_{jk}^{l}$ represents the weight value of the data, *l* denotes the number of layers, *j* stands for the *j*-th neuron, *k* refers to the *k*-th neuron, $a_{j}^{l}$ indicates the weight of a neuron, and $b_{j}^{l}$ represents the bias. The neural network uses the gradient descent algorithm to optimize the value of a single parameter. The parameter update calculation is as follows:
  $$\theta =\theta_{1}-\eta \Delta J(\theta )$$ (4)
  In (4), *θ*_*1*_ refers to the parameter of the last neuron, *J(θ)* refers to the loss function, and *η* stands for the learning rate. When the algorithm is propagated backward, the chain rule of derivatives is adopted, then the derivative of a point *(x*, *y)* can be obtained:
  $$\frac{\text{dz}}{dx}=\frac{dz\cdot dy}{dy\cdot dx}$$ (5)
  Then (5) is generalized to vector form as:
  $$\Delta_{x}{}^{z}={\left(\frac{\partial y}{\partial x}\right)}^{T}\Delta_{y}{}^{z}$$ (6)
  In (6), *Δ*_*x*_^*z*^ and *Δ*_*y*_^*z*^ are the vector values of points *(x*, *y)*, *z* stands for the propagation distance, and *T* refers to the propagation time. Each layer’s information can be reversed from the final loss function continuously using the chain rule, and a smaller storage cost can be used in exchange for an increase in speed. The commonly used loss function is the MSE (Mean Square Error) loss function. The lower the value of this function, the better the model fits in the training set, and the better the effect. The equation of the MSE loss function is:
  $$RMSE=\frac{1}{N}{\sum_{i=1}^{N}\left(Y_{i}-y_{\theta }(x_{i})\right)}^{2}$$ (7)

### Experimental design and material planting

The experiments are in the fields, and five lettuce varieties are tested. The detailed information is shown in Table 1. The tested soil is yellow-brown soil with a total NC (Nitrogen Content) of 0.140%. The total soil NC for the second season planting is 0.168%. The test fertilizer is urea with an NC of 46.4%, produced by Shaanxi Weihe Heavy Chemical Co., Ltd. The type of phosphate fertilizer applied is superphosphate; the application rate is 375 kilogram/hectare. The effective superphosphate content is more than 12%, produced by Changzhou Wunong Agricultural Materials Co., Ltd. The type of potash fertilizer applied is plant ash, and the application rate is (soil: plant ash = 15:1). The plastic flower pots with a diameter of 17.9cm and a height of 16cm are chosen, loading 2kg of air-dried soil through a 0.5cm sieve. After sowing, the seedlings are transplanted to the field when they grow to 5–6 leaves. The experiment adopts a two-factor randomized block experiment, with five planting density levels and four nitrogen fertilizer application levels. Nitrogen fertilizer is applied at the sowing stage, seedling stage, rosette stage, and heading stage with 50%, 10%, 20%, and 20%, respectively. The sowing method is drill seeding, and the row spacing is 30cm. Besides, 80% of samples are used for estimation model construction and model verification, and the remaining 20% are used for model verification.

**Table 1:** Differential classification of different Chinese cabbage varieties.

Numbering	Variety	Subclass
A	Italian lettuce	Rome lettuce
B	Purple Romaine lettuce	Rome lettuce
C	Butterhead lettuce	Looseleaf lettuce
D	Dong Fang Han Si-518 lettuce	Looseleaf lettuce
E	Purple leaf lettuce	Looseleaf lettuce

### Parameter measurement and image acquisition

1. Parameter measurement: the TN (Stem Number) in the seedling stage, rosette stage, and heading stage is manually investigated. Twenty Chinese cabbage plants are sampled from each experimental block. The leaf area is measured using the length-width coefficient method, and the LAI (Leaf Area Index) is calculated. The samples are separated according to organs and dried at 105°C for 30 minutes and dried again at 80°C until constant weight. The DW (Dry Weight) of the above-ground part is measured [27]. The crop samples of different growth stages are divided into stems and leaves, dried, and ground. Then, 0.25g of the ground samples are weighed, and the NC of the samples is measured by the Kjeldahl method [28].
2. Image acquisition: Chinese cabbage canopy images are acquired five times in the seedling stage and once every three to seven days in the rosette stage and heading stage, from 8 a.m. to 9 a.m. when the light is softer. The wireless image acquisition equipment designed by the research team is utilized. An ordinary smartphone is connected to a digital camera (NEX-5R, Sony, Japan) via WiFi, and the smartphone is employed to control the camera to acquire the crop canopy images vertically or the drone to acquire images vertically.

### Construction of Chinese cabbage nitrogen model

The ExG+Ostu method is adopted to remove the background of the field [29]. The ratio of the Chinese cabbage pixel number to the total number of pixels represents the CC (Canopy Cover). The color feature extraction calculation [30] is as follows:

$$NRI=\frac{R}{R+G+B}$$ (8)

$$NGI=\frac{G}{R+G+B}$$ (9)

$$NDI=\frac{R-G}{R+G+0.01}$$ (10)

GMR=G−R (11)

The texture feature extraction [31] is calculated as follows:

$$F_{crs}=\frac{1}{m\times n}\sum_{i=1}^{m}\sum_{j=1}^{m}s^{k}$$ (12)

$$F_{\text{con}}=\frac{\sigma }{\sigma_{4}^{1/4}}$$ (13)

$$F_{lin}=\frac{\sum {}_{i=1}^{m}\sum {}_{i=1}^{m}P_{Dd}(i,j)\text{cos}[(i-j)\frac{2\pi }{n}]}{\sum {}_{i=1}^{m}\sum {}_{i=1}^{m}P_{Dd}(i,j)}$$ (14)

The structure feature extraction [32] is calculated as follows:

$$SSM=k(x,t_{s})=\Delta (\frac{\Delta I(x,t_{s})}{\left|\Delta I(x,t_{s})\right|})$$ (15)

The data are divided into two datasets for modeling and model verification, including the actual measured DW, LAC, SN, CC, and eight feature indicators extracted from the images [33]. The SPSS 24.0 software is employed to analyze the correlation between image feature parameters and agricultural parameters. Image feature values with better correlation with agricultural parameters are filtered out. The multiple stepwise regression method is used to establish the predictive model of agricultural parameters and verify the pros and cons of the model based on R^2^ (Coefficients of Determination of Models) and RMSE (Root Mean Square Error). R^2^ and RMSEP (Root Mean Square Error of Prediction) describe the model’s stability and the average deviation between the measured value and the actual value, and REP (Root Error of Prediction) can evaluate the prediction accuracy of the model.

### Population quality evaluation model

The number of Chinese cabbages in the field is obtained using image analysis technology. Here, the number of Chinese cabbage seedlings in the field are classified into six levels. As shown in Fig 3, the population is divided into low density, high density, and suitable density according to the number of detected Chinese cabbage seedlings. Furthermore, the population is divided into six levels; level 1 indicates severely insufficient seedlings, level 2 indicates insufficient seedlings, level 3 indicates moderately insufficient seedlings, level 4 indicates moderately excessive seedlings, level 5 indicates excessive seedlings, and level 6 indicates severely excessive seedlings.

**Fig 3:** Population basic seedling classification.

The Chinese cabbage population’s quality in different periods is closely related to DW, LAI, TN, and NC. The population is divided into 13 levels through four K-Means Clustering algorithm, as shown in Fig 4. First, the population is classified into high yield, middle yield, and low yield according to the final yield. Second, the middle and low yield populations are classified into large and small populations according to DW and LAI. Third, the large and small populations are classified into two categories: nitrogen deficiency and no nitrogen deficiency according to NC. Finally, according to DW/TN and LAI/TN, the nitrogen-deficient plants are classified as strong individuals and weak individuals.

**Fig 4:** Population quality classification process in different periods.

According to the two-year cultivation experiments and the results of previous works, DW, LAI, TN, NC, and their derived agricultural parameters are selected as the model input. Here, the measured DW, LAI, TN, NC, DW/TN, LAI/TN, NC/TN, NC/DW are used to mark the population level, as shown in Fig 5. The image feature values of the above eight measured indicators and the eight simulated indicators are used as the input to construct the BPNN model for population quality judgment. The ANN (Artificial Neural Network) toolbox of MATLAB 2018b is called. The transfer function between the input layer and the hidden layer is set to the tangent sigmoid function tansig. The transfer function between the hidden and output layers is set to the logarithmic sigmoid function LogSig. The Levenberg-Marquardt backpropagation algorithm is adopted to ensure the network’s rapid convergence, and the dynamic factor is set to 0.01.

**Fig 5:** Structure of population quality evaluation BPNN model.

## Results and discussion

### Image feature value analysis

As shown in Fig 6, the vegetation extraction method proposed above can successfully extract the samples of different growth stages from the farmland. The six image features of the lettuce population can be extracted from the segmented field image. Fig 7 shows the results of image feature values and agricultural parameters. Results demonstrate that some image feature values have extremely significant correlations with agricultural parameters. The two indicators GMR and NGI have the best correlation with NC in lettuce. Besides, the correlation coefficients for different growth stages reach 0.70 or more. CC has a significant correlation with DW, LAI, and TN in the seedling and rosette stages. However, its correlation with the agricultural parameters in the heading stage is not significant. The correlation between the four feature values of Fcrs, Fcon, Ftin, and SSM and the three agricultural parameters of DW, LAI, and TN at the booting stage are all above 0.70.

**Fig 6:** Performance comparison results of different algorithms.

**Fig 7:** Correlation results of image feature values and agricultural parameters. Note: DW refers to the dry weight of the above-ground portion of the crop, TN represents the number of shoots in the field, LAI is the leaf area index, NC is the leaf area index, SS, RS, and HS stand for the seedling stage, rosette stage, and heading stage, respectively.

### Results of the single indicator estimation

As shown in Fig 8, CC positively correlates with the four agricultural indicators of DW, LAI, TN, and NC. CC is exponentially related to the three agricultural parameters of DW, LAI, and NC. The R^2^ values at different levels of nitrogen fertilizer application are 0.7446–0.8121, 0.8346–0.9489, and 0.8531–0.9072, respectively. TN increases first and then decreases with the increase in CC, and the correlation coefficient is between 0.3626 and 0.4558.

**Fig 8:** Cumulative correlation between each indicator and nitrogen.

As shown in Fig 9, the color feature value GMR is positively correlated with the four agricultural parameters. GMR is exponentially correlated with DW, LAI, and NC. The correlation coefficients at different nitrogen levels are 0.8636–0.8899, 0.6316–0.9119, and 0.7054–0.8857, respectively. TN first increases and then decreases with the increase in GMR, and the correlation coefficient is between 0.2924–0.4166. The fitting results of other color features are lower than GMR, and the correlation coefficient R^2^ is lower than GMR. The simulation results of texture feature and morphological feature on various agricultural parameters are not as good as CC and GMR, and the correlation coefficient does not exceed 0.5.

**Fig 9:** Correlation between image color features and various indicators.

### Multiple regression analysis

Fig 10 and Table 2 demonstrate the estimation models of DW, LAI, TN, and NC established by the multiple stepwise regression method and their prediction effects. The four models established have excellent predictive effects on DW, LAI, TN, and NC, and all have higher R^2^ values and lower RMSEP and REP values. The R^2^ value for predicting the four agricultural parameters in the model construction dataset ranges from 0.77 to 0.91, and the REP value ranges from 15.46% to 22.53%; the R^2^ value of the validation dataset ranges from 0.72 to 0.85, and the REP value ranges from 17.31% to 21.26%.

**Fig 10:** Estimation effects of multiple regression model on DW, LAI, TN, and NC.

**Table 2:** Estimation effects of the multiple regression model.

Modeling	Modeling-RMSEP	Verification-RMSEP
DW	883.89	853.16
LAI	0.43	0.55
TN	103.65	119.37
NC	12.21	12.86

Fig 11 displays the test results of the agricultural parameter prediction model established by the SMLR (Syngeneic Mixed Lymphocyte Reaction) method. The model’s prediction error will become larger as the nitrogen application rate increases. The prediction errors of the three agricultural parameters of DW, LAI, and NC increase with the increase in the measured values and the advancement of the fertility process. The error of TN is the largest in the rosette stage.

**Fig 11:** The relationship between the predicted and actual values of agricultural parameters at different nitrogen levels.

### Relationship between parameters and output

As shown in Fig 12, at different levels of nitrogen fertilizer application, the final yield of lettuce increases first and then decreases with the increase in planting density. When the density is between 1.8 million plants per hectare and 2.8 million plants per hectare, the yield will be higher; otherwise, too large or too small density is not conducive to high yield.

**Fig 12:** The correlation between planting density and yield.

As shown in Fig 13, DW, LAI, TN, and NC of the high-yield population in the seedling stage are the principal indicators reflecting the population’s size and nutritional status. Results suggest that the four agricultural parameters of the seedling stage and the lettuce’s final yield show a trend of first decreasing and then increasing. The high-yield population in the seedling stage has DW of 550–800 kilogram/hectare, LAI of 0.8–1.2, NC of 23–28 kilogram/hectare, and TN of 4.7–5.8 million/hectare.

**Fig 13:** The relationship between agricultural parameters and output in the seedling stage.

As shown in Fig 14, the relationship between the four agricultural parameters of DW, LAI, TN, and NC and the final yield is similar to that of the wintering period, all showing a trend of increasing first and then decreasing. The high-yield population in the rosette stage has a DW of 3500–5500 kilogram/hectare, LAI of 3.9–4.5, NC of 90–120 kilogram/hectare, and TN of 10–13 million/hectare.

**Fig 14:** The relationship between agricultural parameters and output in the rosette stage.

As shown in Fig 15, the four agricultural parameters of DW, LAI, TN, and NC at the heading stage also show a trend of first increasing and then decreasing. However, the trend of NC and yield is not apparent. The high-yield population in the heading stage has a DW of 5500–6500 kilogram/hectare, LAI of 6.4–6.7, NC of 120–150 kilogram/hectare, and TN of 5–5.8 million/hectare.

**Fig 15:** The relationship between agricultural parameters and output in the heading stage.

### Population feature evaluation

As shown in Fig 16, the seedling stage population evaluation is based on the basic seedling number. The evaluation aims to determine whether the basic seedling number is reasonable. The accuracy of the evaluation result is affected by the intelligent detection result of lettuce. As the lettuce seedling density increases, the detection error will increase, and the basic seedlings significantly impact the monitoring accuracy. The clustering result suggests that the population of basic seedlings less than 1.35 million per hectare is roughly classified as level 1; that between about 1.35 million and 1.8 million per hectare is classified as level 2; that between about 1.8 million and 2.25 million per hectare is classified as level 3; that between about 2.25 million to 2.70 million per hectare is classified as level 4; that between about 2.70 million and 3.15 million per hectare is classified as level 5, and that above 3.15 million per hectare is classified as level 6. The population is divided into six levels.

**Fig 16:** Population quality evaluation results in the seedling stage.

### Population quality evaluation

As shown in Fig 17, independent samples are utilized to evaluate the constructed quality evaluation model of lettuce populations. The model that directly uses color feature values as input parameters is set as CI, and the DW, LAI, and LAI estimated by image analysis technology are set. The model in which TN and NC and their derivatives are used as input parameters is PI. The model evaluates the results of the lettuce population in different periods. In the three growth stages, the average R^2^ value of the population quality evaluation using the PI model is 0.83, and the average RMSE is 1.56. The CI model’s evaluation error is comparatively large, the R^2^ value does not exceed 0.3, and the seedling stage RMSE is as high as 4.85, showing that the PI model’s evaluation effect is better and can evaluate the population quality. The predicted value of the rosette stage PI model is mostly concentrated around 1:1.

**Fig 17:** BPNN model evaluation results of population quality in different periods.

In contrast, the predicted value of the CI model is scattered, and the value of the PI model is much higher than the CI model. The quality of the heading stage population and the actual value of population quality is 1: 1. The outcome is similar to the wintering period and jointing period, but the R^2^ value is lower.

## Conclusions

The Chinese cabbage population is monitored since the seedling stage. Computer vision technology is employed to acquire agricultural parameters that can exhibit the Chinese cabbage population quality. An estimation model of LAI, DW, TN, and NC of plants in different periods during winter is established based on digital image technology characteristics. This model can accurately estimate NC in the Chinese cabbage population. Besides, a population quality evaluation model is constructed based on the intelligent acquisition of agricultural parameters, combined with neural network technology, to explore the relationship between population agricultural parameters and output in different periods. The classification standards for Chinese cabbage population quality are formulated, and an evaluation model for Chinese cabbage population quality is constructed. This model can evaluate the population quality of Chinese cabbage in different periods. The average R^2^ value of using the model to evaluate population quality is 0.83, and the average RMSE is 1.56, which further confirms that the proposed model has high accuracy and small errors. It can provide some research ideas for crop cultivation in modern agriculture. Referring to Dr. Sun’s research, the research on Chinese cabbage can be further extended to other fields [34]. Although digital images and intelligent algorithms are applied to crop nutrition monitoring, several shortcomings are found in the investigation process. First, there are many image processing methods, such as noise reduction and resolution improvement, which can effectively improve recognition accuracy. Second, deep learning algorithms can be used for digital image modeling, improving the learning depth of the data. These two aspects will be explored in-depth in future works to improve the model continuously.

## Supporting information

S1 Data (XLSX)
